The article "Assessment of Tumor Cells in a Mouse Model of Diffuse Infiltrative Glioma by Raman Spectroscopy" was published in 2014. Journal: Biomed Res Int.

# Assessment of Tumor Cells in a Mouse Model of Diffuse Infiltrative Glioma by Raman Spectroscopy

**DOI:** 10.1155/2014/860241

**Published:** 2014-08-27

**Authors:** Kuniaki Tanahashi, Atsushi Natsume, Fumiharu Ohka, Hiroyuki Momota, Akira Kato, Kazuya Motomura, Naoki Watabe, Shuichi Muraishi, Hitoshi Nakahara, Yahachi Saito, Ichiro Takeuchi, Toshihiko Wakabayashi

**Affiliations:** ^1^Department of Neurosurgery, Nagoya University School of Medicine, 65 Tsurumai-cho, Showa-ku, Nagoya 466-8550, Japan; ^2^Division of Epigenomics and Molecular Oncology, Aichi Cancer Center Research Institute, Japan; ^3^Renishaw, Raman Group, Japan; ^4^Department of Quantum Engineering, Nagoya University School of Engineering, Japan; ^5^Department of Computer Science/Scientific and Engineering Simulation, Nagoya Institute of Technology, Japan

## Abstract

Glioma of infiltrative nature is challenging for surgeons to achieve tumor-specific and maximal resection. Raman spectroscopy provides structural information on the targeted materials as vibrational shifts. We utilized Raman spectroscopy to distinguish invasive tumors from normal tissues. Spectra obtained from replication-competent avian sarcoma-(RCAS-) based infiltrative glioma cells and glioma tissues (resembling low-grade human glioma) were compared with those obtained from normal mouse astrocytes and normal tissues. In cell analysis, the spectra at 950–1000, 1030, 1050–1100, 1120–1130, 1120–1200, 1200–1300, 1300–1350, and 1450 cm^−1^ were significantly higher in infiltrative glioma cells than in normal astrocytes. In brain tissue analysis, the spectra at 1030, 1050–1100, and 1200–1300 cm^−1^ were significantly higher in infiltrative glioma tissues than in normal brain tissues. These spectra reflect the structures of proteins, lipids, and DNA content. The sensitivity and specificity to predict glioma cells by distinguishing normal cells were 98.3% and 75.0%, respectively. Principal component analysis elucidated the significance of spectral difference between tumor tissues and normal tissues. It is possible to distinguish invasive tumors from normal tissues by using Raman spectroscopy.

## 1. Introduction

Glioma is the most common and lethal primary brain tumor [1]. Current treatment regimens, including surgery followed by chemoradiotherapy, have improved the outcomes of patients with malignant glioma (MG) to some extent [2]. However, those improvements have not shown sufficient impact, and long-term control of the disease is rarely achieved.

In glioma surgery, the extent of tumor resection is one of the main determinants of prognosis. However, due to the infiltrative nature of gliomas, it is often challenging for surgeons to determine the resection border for tumors that appear in normal brain. Several useful modalities have been developed for safe and maximum tumor resection, such as neuronavigation, electrophysiological monitoring, intraoperative magnetic resonance imaging (MRI), and fluorescent-guided surgery; unfortunately, these modalities and technologies are not fully satisfactory. In an attempt to achieve tumor-specific resection that leads to a more favorable outcome, new methods to detect tumor boundaries more precisely, and in real-time during surgery, must be developed.

The article "Assessment of Tumor Cells in a Mouse Model of Diffuse Infiltrative Glioma by Raman Spectroscopy" was published in 2014. Journal: Biomed Res Int.

Raman spectroscopy, which is based on vibrational spectroscopic techniques, is used to derive the chemical structure of substances [3]. Most of the photons of incident light that strike a given molecule are elastically scattered with the same energy, but a small amount of photons (only 1 per 10 million) are inelastically scattered with different vibrational frequencies [3]. This vibrational shift, which is manifested as a wavenumber shift or Raman shift, is a characteristic of specific molecules or chemical bonds and thus can be used to provide structural information on the targeted materials [3].

Although Raman spectroscopy is predominantly used for chemical analysis [4], its unique properties can also be applied to biological analyses [3–5]. Specifically, it can detect chemical characteristics of biomaterials at the molecular level, and because the excitation light has weak energy, it is not destructive for tissue specimens [3, 4]. High spatial resolution is achieved with measurement spots of less than 1 *μ*m [3]. The signal distortion from water is minimum compared with infrared spectroscopy, an alternative method that yields complementary information [3].

We hypothesized that it might be possible to distinguish invasive tumors from normal tissues using Raman spectroscopy. Therefore, spectra obtained from mouse infiltrative glioma cells and tissues were compared with those from normal mouse astrocytes and brain tissues. An advantage of our approach is that the intrinsic and invasive mouse glioma model recapitulates many features of human gliomas, in contrast to previous studies of artificial well-demarcated xenografts [6]. Our data provide proof-of-concept that Raman spectroscopy can discriminate infiltrated areas from normal brain regions. This suggests that the technique could be a potential diagnostic tool in glioma surgery that enables in situ and real-time tissue assessments.

## 2. Materials and Methods

### 2.1. Establishment of a Mouse Model of Infiltrative Glioma Using the RCAS/tv-a System

We used a replication-competent avian sarcoma and leukemia virus long terminal repeat with splice acceptor (RCAS)/tumor virus A (tv-a) system as previously described [7, 8]. The protocols for animal experiments were approved by the Animal Experiment Committee of Nagoya University. Briefly,* platelet-derived growth factor subunit B (PDGFB)* was used to initiate an infiltrative glioma that resembles WHO Grade II human oligodendroglioma histologically. The histology of oligodendroglioma typically shows mild to high populated round cells often referred to as “fried egg” cells. The RCAS-PDGFB plasmid, which contains full-length, wild-type human* PDGFB*, was a gift from Eric C. Holland (Memorial Sloan-Kettering Cancer Center). DF-1 cells, immortalized chicken fibroblasts (American Type Culture Collection), were grown as producer cells in Dulbecco's modified Eagle medium (DMEM) containing 10% fetal bovine serum (FBS), 100 mg/mL streptomycin, and 100 IU/mL penicillin in a 5% CO_2_ humidified incubator at 37°C. RCAS vectors were transfected into DF-1 cells using FuGene6 (Roche, Basel, Switzerland) and allowed to replicate in culture. DF-1 cells (1 × 10^5^ cells in 1-2 *μ*L of PBS) were injected into the right frontal lobe of Gtv-a mice, which are transgenic for tv-a under the control of the glial fibrillary acid protein promoter, at the time of birth from an entry point just anterior to the coronal suture of the skull using a 10-*μ*L glass syringe.

The article "Assessment of Tumor Cells in a Mouse Model of Diffuse Infiltrative Glioma by Raman Spectroscopy" was published in 2014. Journal: Biomed Res Int.

### 2.2. Single Cell Culture

Gtv-a mice harboring gliomas were euthanized with CO_2_ inhalation. The tumors were aseptically removed and enzymatically dissociated with trypsin-EDTA for 15 min at 37°C. The digestion was stopped with DMEM containing 10% FBS. After trituration with a pipette, single cells were washed, plated, and cultured in DMEM containing 10% FBS, 100 mg/mL streptomycin, and 100 IU/mL penicillin at 37°C in a humidified 5% CO_2_ atmosphere. Normal mouse astrocytes were prepared from the primary mixed glial cell cultures of newborn ICR mice (SLC, Shizuoka, Japan), as described previously [9]. Astrocytes were purified from the primary mixed glial cell cultures by three to four repetitions of trypsinization and replating. Cultures were maintained with DMEM supplemented with 10% FBS and 5 *μ*g/mL of bovine insulin. The astrocytes were grown to confluency, and the medium was exchanged every three days.

### 2.3. Raman Spectroscopy of Glioma Cells and Astrocytes

Cultured glioma cells and astrocytes were harvested and 1 × 10^4^ cells were seeded onto the quartz plates at the center of 35-mm dishes. The dishes were then filled with media after attaching the seeded cells on the plates. After culturing for two to three days, the cells were submitted for Raman analysis. Media were removed and replaced by saline prior to examination to avoid distortion of Raman spectra by phenol red contained in the media.

The article "Assessment of Tumor Cells in a Mouse Model of Diffuse Infiltrative Glioma by Raman Spectroscopy" was published in 2014. Journal: Biomed Res Int.

Spectral data were collected with an inVia Raman microscope (Renishaw, Gloucestershire, UK) using an excitation laser of 532 nm, a ×63 objective lens, and a 1800 lines/mm grating setting. Measurements of four accumulations were taken. The laser power was 2.25 mW and exposure time was 10 × 4 s per spectrum. By using Raman processing software, each spectrum was background corrected by subtracting the solvent background, normalization of the phenylalanine band, and cosmic ray removal. Spectra not covering the “fingerprint” range from 580 to 1,800 cm^−1^ were removed. In the cell analysis, 40 spectra from 2 normal astrocytes and 58 spectra from 4 glioma cells were recorded.

### 2.4. Raman Spectroscopy of Mouse Brain Tissues

Gtv-a mice were euthanized as described above and the brains were sliced coronally at the tumor location with 1-mm thickness. The sliced brain tissues were dipped in Hanks' Balanced Salt Solution (Life Technologies, Carlsbad, CA) and kept on ice. The sample tissues were washed with saline before examination to prevent distortion of signals by phenol red. Samples were placed on quartz plates at the center of 35-mm dishes, which were then filled with saline to prevent dehydration.

A total of 123 spectra were collected randomly from 6 brain tissues. The laser power was 45 mW and exposure time was 10 × 4 s per spectrum. Mapping of mouse brain slices was performed using the same laser and power. Raman images of 264 (12 × 22) spectra were recorded with a step size of 300 *μ*m, 7 s dwell time to bleach autofluorescence, and 1 × 3 s exposure time per spectrum using a ×63 water-immersion objective. Spectral processing after the measurement was done in the same manner as described above.

After the measurement, adjacent sites of the brain tissues were fixed in 4% paraformaldehyde (Wako, Osaka, Japan) and embedded in paraffin using a Tissue-Tek rotary tissue processor (Sakura Finetek, Tokyo, Japan) and 5-*μ*m sections were cut with a microtome (Leica Microsystems, Wetzlar, Germany). The sections were stained with hematoxylin and eosin (H&E) for confirmation of the tumor locations. As this is an infiltrative tumor, there is no clear margin. Histologically, we defined the hypercellular area that consisted of “fried egg” cells as the tumor area and the area with no/few tumor cells as the normal area, with the borderline area located between these two areas.

### 2.5. Statistical Analysis

The obtained spectra were standardized to have zero mean and unit variance before proceeding with statistical analysis. Statistical significance of the difference between tumor and normal samples was measured for each spectrum using the *P* value and false discovery rate (FDR) based on* t*-statistics (FDR was computed by permutation label permutation).

The article "Assessment of Tumor Cells in a Mouse Model of Diffuse Infiltrative Glioma by Raman Spectroscopy" was published in 2014. Journal: Biomed Res Int.

Linear logistic regression analysis was conducted to compute the tumor probability of each location, where the output from the model ranges between 0 and 1 and values greater than 0.5 were considered as tumor (positive) whereas those lower were regarded as normal (negative). The data from borderline areas were excluded from the tumor predictions.

Since the number of variables, that is, the number of wavenumber steps within the measured range 580 to 1,800 cm^−1^, was far more than the number of the samples, a certain form of parameter restriction was required when the model was fitted. We used L2 penalization (penalizing the squared norm of the parameter vector). The amount of penalization was objectively determined by leave-one-out cross-validation within the sample training set.

In order to estimate the out-of sample performance of the tumor probability predictions, we used what we termed “leave-cell-out” and “leave-mouse-out” cross-validation for cell and brain tissue data, respectively. Specifically, this means that when the tumor probability of a sample in a certain cell is predicted, all the samples taken from that cell are omitted when the model is fitted.

To visualize the two identified clusters (brain tumor and normal brain), principal component analysis (PCA) was applied to the spectral data and 3D ellipsoids representing the covariance structure of each cluster were drawn in the 3D plots of the first 3 principal components.

All the statistical analyses except the 3D PCA plot (which was generated by JMP ver.9.0) were performed using R^23^.

## 3. Results

### 3.1. Raman Spectrum of Glioma Cells and Normal Astrocytes

We first evaluated the difference in Raman scattering spectra between glioma cells and normal astrocytes (Figure 1(a)). As shown in Table 1, the spectra at 950–1000, 1050–1100, 1120–1130, 1120–1200, 1200–1300, and 1300–1350 cm^−1^ are derived from chemical structures C–C (protein), C–C (lipid), C-C (lipid), C–C/C–N (protein), amide III, and C–H_2_ (lipid), respectively. The spectra around 1030, 1100, and 1450 cm^−1^ are derived from O–P–O (nucleic acid), C–H (phenylalanine), and C–H_2_ twist (lipid). These Raman signals were significantly higher in glioma cells than in normal astrocytes (Figures 1(b) and 1(c)) and reflect proteins, lipids, and DNA content.

### 3.2. Raman Spectrum of Infiltrative Glioma in the Mouse Brains

We next investigated whether Raman spectroscopy distinguished glioma tissues from normal brain tissues in an ex vivo infiltrative glioma mouse model.* PDGFB*-induced glioma models are distinct from xenograft models in which human glioma cells are implanted in the brain of immune-deficient mice. This is since xenografts have high tumor cellularity and a clear border between the tumor tissue and the normal brain and also distort the normal tissue structure. In the current study, we utilized a model of WHO Grade II glioma, specifically oligodendroglioma, a clinical stage at which it is often difficult to distinguish tumors from normal brain tissues during surgery. Similar to the cell analysis, the average spectra in the six brains at 1030 (C–H; phenylalanine), 1050–1100 (C–C; lipid), 1100 (O–P–O; DNA), and 1200–1300 cm^−1^ (amide III) were significantly higher in glioma tissues than in the normal brains. Representative images of H&E staining and 3D plots of PCA were shown in Figure 2(c). The clusters of tumor (red ellipsoids) were separated from those of normal (blue ellipsoids), which supported the significance of spectral difference between tumor tissues and normal tissues.

The article "Assessment of Tumor Cells in a Mouse Model of Diffuse Infiltrative Glioma by Raman Spectroscopy" was published in 2014. Journal: Biomed Res Int.

### 3.3. Tumor Prediction

Predictions of tumor probability were made (see Methods). The outputs from the model were described as blue dots within the range between 0 and 1, and values greater than 0.5 were considered as tumor (positive; green dots on the position of 1), whereas those lower were regarded as normal (negative; green dots on the position of 0). True tumors and normals were described as red dots on the position of 1 and the position 0, respectively. The sensitivity and specificity were 98.3% and 75.0%, respectively (Figure 3(a)). While the accuracy of tumor prediction probability in brain tumor tissues was not as robust as it was in cells, the specificity was still high (76.4%, Figure 3(b)).

### 3.4. Raman Chemical Imaging in Tissues

Based on our findings that major differences in Raman signals between tumor and normal brain reflected lipid contents, we sought to obtain Raman chemical image in tissues. The process for mapping the whole slice is long, and we were unable to locate the tumor region before the procedure. Thus, we randomly mapped four regions and used H&E staining of an adjacent brain slice to retrospectively identify the one region containing tumor material. A representative map image and the adjacent H&E section are shown in Figure 4; a high signal (red) is evident in the region containing the tumor.

## 4. Discussion

Raman spectroscopy is increasingly applied for histopathological analyses. Using this technique, cancers of cervix, lung, breast, prostate, and skin could be distinguished from normal tissues [10–15]. Raman spectroscopy has also been applied to diagnosis of experimental glioma [16–19]. Raman spectroscopy has several advantages over conventional approaches to histopathological diagnosis. In contrast to H&E staining, it requires no pretreatment, it takes less than a minute to examine each spot, and it is not destructive to the samples. Furthermore, with the use of color mapping, it enables high-resolution images to be produced. Although infrared spectroscopy gives information complementary to that of Raman spectroscopy, infrared signals are susceptible to interference from strong water absorption and the spatial resolution is lower compared to Raman spectroscopy [3–5, 20, 21].

The article "Assessment of Tumor Cells in a Mouse Model of Diffuse Infiltrative Glioma by Raman Spectroscopy" was published in 2014. Journal: Biomed Res Int.

Previously, Ji et al. delineated human glioma xenografts in mice using Raman spectroscopy [22]; they utilized abundant proteins in glioma tissues and lipid-rich normal white matter. However, their model did not recapitulate the true composition and context of infiltrative glioma. For example, the implanted tumor was not derived from native brain tissue and the extraneous tumor distorted the surrounding normal tissues. In our study, we instead used an infiltrative glioma mouse model, which more closely reflects the nature of infiltrative glioma that has an indistinct margin [7, 8].

We showed significant differences in Raman spectra between mouse glioma cells and normal astrocytes and between mouse infiltrative glioma tissues and normal brain tissues. In the cell analysis, the spectra at 950–1000, 1050–1100, 1120–1130, 1120–1200, 1200–1300, and 1300–1350 cm^−1^ and the peaks around 1100, 1030, and 1450 cm^−1^ were higher in glioma cells than in normal astrocytes. Those peaks are derived from the chemical structure of DNA, proteins and lipids as described in Table 1. Several biologically significant peaks exist in those regions as previously reported [23].

In the tissue analysis, we examined fresh brain tissue sections but not frozen ones. Spectra at 1030, 1050–1100, 1100, and 1200–1300 cm^−1^, which are consistent with the peaks of C–H (phenylalanine), C–C (lipid), O–P–O (DNA), and protein, respectively, were higher in glioma tissues than in normal brain tissues. This is reasonable, since tumor cells frequently harbor amplified genes and other chromosomal aberrations, overexpression of proteins, and hypermetabolism of lipids, along with their increased mitotic activity [24].

We could not apply the prediction algorithm developed during the cell analysis to the tissue analysis. This is due to differences in optical properties in each setting. In the tissue analysis, near infrared excitation is optimal for reducing competing fluorescence from the tissue itself, for avoiding the noise generated by water in tissues, and for optimal penetration of the surface of tissues. By contrast, in the cell analysis, near infrared was not applicable due to the strong noise from the quartz plate [11, 25].

The article "Assessment of Tumor Cells in a Mouse Model of Diffuse Infiltrative Glioma by Raman Spectroscopy" was published in 2014. Journal: Biomed Res Int.

A cell contains nuclei and cytoplasmic organelles, and a brain tissue consists of cortex, white matter, and basal ganglia. Indeed, a previous study showed that porcine white matter contained more lipid than gray matter [26]. In this study, we standardized the heterogeneity by collecting spectra from adequate amount of spots distributed on the entire surface.

In the tissue analysis, the difference between tumor spectra and normal brain spectra was less distinct. We speculate that this is because each examined spot included more heterogeneous components of the tissues than those of single cells. Moreover, recent works have demonstrated that the peritumoral tissue, even in the absence of clear neoplastic infiltration, presents biological alterations suggestive of a precancerous condition [27–30]. One possible improvement is to enhance the spectral signature in order to clearly detect tumors. Surface-enhanced Raman scattering (SERS) nanoparticles have been used as molecular imaging contrast agents in conjunction with Raman spectroscopy [31]. This enabled the delineation of contrast-enhanced tumors distinctly before and during resection of xenograft gliomas in mice. SERS nanoparticles accumulated and were retained in the tumor due to a compromised blood-brain barrier [32]. However, this particular application is limited to contrast-enhanced tumors, and SERS nanoparticles would not be distributed into nonenhanced tumors such as low-grade glioma, in which the blood brain barrier is not disrupted. Even in high-grade glioma, tumor cells infiltrate the surrounding tissue without contrast enhancement [33]. Other groups have detected biomarkers in serum using immunoassay in combination with SERS, an approach that is useful for tumors that release specific biomarkers into the serum [34, 35].

In other studies, fiber-optic endoscopic probes have been used in conjunction with Raman spectroscopy for the analysis of esophageal and gastric cancer in vivo and ex vivo [36, 37]. This is a promising tool for intraoperative diagnosis during endoscopic resection of esophageal intramucosal cancer. If a similar probe could be developed for brain tumor surgery, surgeons could utilize it to depict the borderlines of infiltrative glioma.

We believe that our study demonstrates that Raman spectroscopy is a promising tool for brain tumor surgery, especially in cases of infiltrative glioma. Further preclinical and clinical studies should be scheduled in order to further substantiate this hypothesis.

The article "Assessment of Tumor Cells in a Mouse Model of Diffuse Infiltrative Glioma by Raman Spectroscopy" was published in 2014. Journal: Biomed Res Int.

## Figures and Tables

**Figure 1:** Raman spectrum of glioma cells and normal astrocytes. (a) Measurement of Raman scattering spectra in glioma cells and normal astrocytes. (b) The difference in Raman scattering spectra between glioma cells (red) and normal astrocytes (blue). (c) Statistical analysis. Statistical significance of the difference between tumor and normal samples was measured for each spectrum using the *P* value (red) and false discovery rate (FDR; blue) based on* t*-statistics (FDR was computed by permutation label permutation).

**Figure 2:** Raman spectrum of infiltrative glioma in the mouse brains. (a) The average spectra in the six brains at 1030 (C–H; phenylalanine), 1050–1100 (C–C; lipid), 1100 (O–P–O; DNA), and 1200–1300 cm^−1^ (amide III) were significantly higher in glioma tissues (red) than in the normal brains (blue). (b) Statistical analysis. Statistical significance of the difference between tumor and normal samples was measured for each spectrum using the *P* value (red) and false discovery rate (FDR; blue) based on* t*-statistics (FDR was computed by permutation label permutation). (c) Representative images of H&E staining and 3D plots of principal component analysis. The clusters of tumor (red ellipsoids) were separated from those of normal (blue ellipsoids), which supported the significance of spectral difference between tumor tissues and normal tissues.

**Figure 3:** Tumor prediction. The outputs from the model were described as blue dots within the range between 0 and 1, and values greater than 0.5 were considered as tumor (positive; green dots on the position of 1), whereas those lower were regarded as normal (negative; green dots on the position of 0). (a) True tumors and normals were described as red dots on the positions of 1 and 0, respectively. The sensitivity and specificity were 98.3% and 75.0%, respectively. (b) While the accuracy of tumor prediction probability in brain tumor tissues was not as robust as it was in cells, the specificity was still high (76.4%).

**Figure 4:** Raman chemical imaging in tissues. (a) A representative map image based on lipid contents. The white arrow indicates high signal of lipids. (b) The adjacent H&E section. The large inset corresponds to the mapping area of (a). (c) The high magnification of the small inset in (b). A high signal (red) in (a) is evident in the region containing the tumor. The border is represented as green area.

**Table 1:** Raman shift corresponding to chemical structure.

Shift (cm^−1^)	Chemical structure
950–1000	C–C (protein, collagen)
1004	phenylalanine
1030	C–H (phenylalanine)
1050–1100	C–C (lipid)
1100	O–P–O (phosphate backbone)
1120–1130	C–C (lipid)
1120–1200	C–C/C–N (protein)
1200–1300	amide III, a-helix, b-sheet
1300–1350	C–H_2_ (lipid), protein, nucleic acid
1450	C–H_2_ (lipid)
